This article has been retracted.

# Transformer 2 alpha homolog is a downstream gene of hypoxia-inducible factor 1 subunit alpha and is involved in the progression of pancreatic cancer

**DOI:** 10.1080/21655979.2022.2079243

**Published:** 2022-05-29

**Authors:** Wenpeng Cao, Shan Lei, Zhirui Zeng, Chaolun Xiao, Baofei Sun, Peng Xie, Yumei Li, Daopeng Luo, Wenfeng Yu

**Affiliations:** a Department of Anatomy, School of Basic Medicine, Guizhou Medical University, Guiyang, Guizhou, China; b Department of Physiology, School of Basic Medicine, Guizhou Medical University, Guiyang, Guizhou, China; c Key Laboratory of Endemic and Ethnic Diseases, Ministry of Education, School of Basic Medical, Guizhou Medical University, Guiyang, Guizhou, China; d Key Laboratory of Medical Molecular Biology, School of Basic Medical, Guizhou Medical University, Guiyang, Guizhou, China

**Keywords:** Pancreatic cancer, hypoxia, transformer2A proteins, hypoxia-inducible factor 1-alpha

## Abstract

Intratumoral hypoxia is a common feature of pancreatic cancer (PC) and also plays a role in its progression. However, hypoxia-regulated signatures in PC are still not completely understood. This study aimed to identify core hypoxia-associated genes and determine their underlying molecular mechanisms in PC cells. Transformer 2 alpha homolog (TRA2A) was found to be an important hypoxia-associated gene, which was upregulated in PC tissues and in PC cells cultured under hypoxia. High TRA2A expression was associated with advanced stage, poor differentiation, and lymph node metastasis. Under normoxic and hypoxic conditions, knockdown of TRA2A both markedly suppressed PC cell proliferation and motility *in vitro* and *in vivo*, as well as activation of the AKT pathway. Hypoxia-inducible factor 1 subunit alpha (HIF1α) upregulated the transcription of TRA2A by directly binding to its promoter. TRA2A showed a co-expression relationship with HIF1α in PC tissues. Overexpression of TRA2A alleviated the pro-inhibitive functions of HIF1α-inhibition on PC cell proliferation and motility under hypoxia. In conclusion, TRA2A is a crucial downstream gene of HIF1α that accelerates the proliferation and motility of PC cells. TRA2A may be a novel and practical molecular target for investigating the hypoxic response of PC cells.

**Abbreviations**: TRA2A, transformer 2A protein; PC, pancreatic cancer; HIF1α, hypoxia-inducible factor 1-alpha; GEO, Gene Expression Omnibus; IHC, immunohistochemical staining.

## Highlights

- TRA2A was upregulated in PC cells under hypoxia.
- TRA2A inhibition reduced PC progression under normoxia and hypoxia.
- TRA2A regulated the AKT pathway in normoxia and hypoxia.
- HIF1α directly regulated TRA2A expression.
- Overexpression of TRA2A reversed the effects of HIF1α knockdown.

## Introduction

As one of the most aggressive malignancies, pancreatic cancer (PC) is the fourth leading cause of cancer-associated death worldwide [1]. Despite multiple advances in PC therapy strategies, the 5-year survival rate of patients remains lower than 6% because of the high incidence of tissue invasiveness and metastasis [2]. Thus, there is an urgent need to delve into the molecular mechanisms regulating the progression of PC, which is beneficial for developing PC therapies.

Hypoxia commonly exists in solid tumors because of excessive oxygen consumption due to rapid cancer proliferation and insufficient vascular supply [3]. Hypoxia has been shown to accelerate PC cell proliferation, metastasis, differentiation, and treatment resistance [4–6]. During hypoxia, hypoxia-inducible elements play immediate and central roles by binding to the promoter and driving the transcription of a series of target genes, thus accelerating vascularization, proliferation, and distant metastasis [4,7]. Cao *et al*. demonstrated that the hypoxia-related gene fucosyltransferase 11 is highly expressed in PC tissues and accelerates metastasis of PC cells by upregulating the expression of pyruvate dehydrogenase kinase 1 [8]. Similarly, Zeng *et al*. indicated that HIF1α regulates hypoxia-induced proliferation and invasion by elevating the expression of YEATS domain-containing protein 2 [9]. Cao *et al*. showed that hypoxic pancreatic stellate cell-derived exosomal miRNAs drive the proliferation and mobility of pancreatic cancer through the PTEN/AKT pathway [10]. However, the hypoxia-regulated network of PC cells remains unclear.

Mammalian homologs of TRA2 possess two different gene paralogs that encode TRA2A and TRA2B proteins [11]. TRA2B is associated with cancer cell survival and therapeutic sensitivity [12–14]. Many studies have shown that TRA2A acts as an oncogene in various cancers [15]. TRA2A is upregulated in glioma cells and drives epithelial-mesenchymal transition [16]. High TRA2A expression is associated with prostate cancer progression [17]. However, the association between TRA2A and hypoxia in PC remains unclear.

In this study, we aimed to identify the biological functions of TRA2A and explore its association with HIF1α in PC cells. We found that TRA2A is a downstream gene of HIF1α and is involved in the proliferation and motility of PC. TRA2A may be a distinct target for suppressing the accelerating role of the hypoxic environment in PC cells.

## Materials and methods

### Bioinformatics analysis

The gene expression matrix (serial number: GSE9350) [18] was accessed from the Gene Expression Omnibus (GEO) database (https://www.ncbi.nlm.nih.gov/gds). Six normoxic and six hypoxic PC samples were identified from GSE9350. A log fold change (FC) >1.0, combined with an adjusted P-value <0.05, was set as the threshold to determine differentially expressed genes. The differentially expressed genes are shown in a volcano plot.

### Cell culture and clinical specimen

The PC cell lines PANC-1 (catalog no: ATCC CRL-1469) and Capan-2 (catalog no: ATCC HTB-80) were purchased from the American Type Culture Collection (ATCC, USA). PANC-1 and Capan-2 cells were cultured at 37°C in 5% CO_2_ in Dulbecco’s modified Eagle medium (DMEM; Thermo Fisher Scientific, USA) containing 10% fetal bovine serum (FBS; Thermo Fisher Scientific, USA). To create a hypoxic microenvironment, PC cells were placed in a three-gas incubator (Thermo Fisher Scientific, USA), and the oxygen concentration was set at 1%. The Affiliated Hospital of Guizhou Medical University provided 48 paired clinical PC samples, collected between January 2019 and December 2020, for this study. The Human Research Ethics Review Committee of Guizhou Medical University approved the application of these clinical samples (approved number: 2022–11), which was performed according to the tenets of the Declaration of Helsinki.

### Cell transfection

Small interfering RNAs targeted against TRA2A (si1-TRA2A and si2-TRA2A) and HIF1α (si-HIF1α), and the corresponding negative control (si-NC) were purchased from Sangon Biotech (Shanghai) Co., Ltd. The sequence of siRNA control was ACGUGACACGUUCGGAGAATT, the sequence of si1-TRA2A was UUGGGAUCUGGAUUUGCCCTT, the sequence of si2-TRA2A was GUUGUGUACAAACUGAGGCTT, and the sequence of si-HIF1α was CAAGUAGCCUCUUUCACAA. The TRA2A-overexpressing plasmid, HIF1α-overexpressing plasmid, and its matched control were acquired from Genechem (Shanghai) Co., Ltd. siRNAs and plasmids transfection process was carried out via Lipo 2000 reagent (Ribobio; ThermoFisher Scientific, USA) based on the manufacturer’s guide.

### Quantitative real-time fluorescence PCR (qRT-PCR)

Total RNA from PC cells and tissues was isolated using TRIzol reagent (Invitrogen, USA). A kit of complete reagent for first-strand cDNA synthesis (Sigma-Aldrich, USA) was used to reverse transcribe mRNAs into cDNAs. The mRNA expression of target genes was determined using KAPA SYBR® FAST reagent (Sigma-Aldrich, USA). β-actin was used as a loading control. The primers used were as follows:

HIF1α forward primer 5′-ATCCATGTGACCATGAGGAAATG-3′, HIF1α reverse primer 5′-TCGGCTAGTTAGGGTACACTTC-3′, TRA2A forward primer 5′- GGTCAGGATCTCGTAGTCCAT-3′, TRA2A reverse primer 5′- CCTCGACCTGGATTTTGATCTTG-3′, β-actin forward primer 5′-CATGTACGTTGCTATCCAGGC-3′, and β-actin reverse primer 5′-CTCCTTAATGTCACGCACGAT-3′.

### Proliferation analysis

The cell proliferation rate was determined using the Cell Counting Kit-8 reagent (Invitrogen, USA). Briefly, the PC cells were seeded into 96-well-plates at a density of 4 × 10^3^ cells/well, followed by culture at 37°C in 5% CO_2_. After 24-hour and 48-hour incubation, the culture medium was replaced, and 10 µL CCK-8 solution was added to each well. The plate was then placed in a 37°C incubator for 2 h. The absorbance was measured at a wavelength of 450 nm.

### Wound healing assay

The PC cells were seeded onto 6-well plates, followed by culture until >95% confluence. A 200 µL pipette tip on the cell monolayer was used to generate a scratch lesion. The cells were then washed three times with PBS and a fresh serum-free medium was added. The status of the wound was monitored using an optical microscope from 0 to 24 h.

### Transwell assay

Each group of PC cells (5 × 10^4^/well) was placed in an FBS-free medium in the upper transwell chamber (Corning Incorporated, USA) pre-coated with Matrigel (Corning Incorporated, USA). Next, 700 µL medium with 10% FBS was placed in the lower chamber. After 24 h, the top chambers were fixed using 4% paraformaldehyde for 15 min and stained with 1% crystal violet for 20 min. A cotton swab was then used to remove non-invading cells from the upper surface. Invasive cells per field were counted using an optical microscope (Thermo Fisher Scientific, USA).

### Western blot

Cells were lysed with RIPA lysis buffer reagent (CapitalBio Technology, Beijing, China) containing 1% proteinase inhibitor PMSF (CapitalBio Technology, Beijing, China) on ice for 30 min. After centrifugation at 13,000 *g* for 15 min, supernatants were collected and quantified using the BCA detection method. Total protein obtained from each sample (30 μg/lane) was separated using 12% SDS-PAGE gel (Thermo Fisher Scientific, USA) and transferred onto PVDF membranes (Millipore, USA). After blocking using 5% BSA, the membranes were incubated with anti-TRA2A (dilution 1:1,000; catalog number: 12,079-1-AP; Proteintech, Wuhan, China), AKT (dilution 1:1,000; catalog number: 60,203-2-Ig; Proteintech, Wuhan, China), p-AKT (dilution 1:1,000; catalog number: 80,455-1-RR; Proteintech, Wuhan, China), PTEN (dilution 1:1,000; catalog number: 22,034-1-AP; Proteintech, Wuhan, China), anti-KI67 (dilution 1:1,000; catalog number: 27,309-1-AP; Proteintech, Wuhan, China), anti-PCNA (dilution 1:1,000; catalog number: 10,205-2-AP; Proteintech, Wuhan, China), anti-HIF-1α (dilution 1:1,000; catalog number: 66,730-1-Ig; Proteintech, Wuhan, China) and anti-β-actin (dilution 1:1,000; catalog number: 66,009-1-Ig; Proteintech, Wuhan, China). After incubation with a horseradish peroxidase-conjugated secondary antibody (dilution 1:5,000; Beyotime, Shanghai, China) for 2 h, the protein bands were visualized using ECL reagent (Affinity, USA). Image Pro-Plus software was used to analyze protein expression, and β-actin was used as a loading control.

### In vivo assay

For the subcutaneously injected model, 10 female BALB/c nude mice were obtained from the Animal Center of Guizhou Medical University (Guizhou, China). After adaptive feeding, 2 × 10^6^ PANC-1 cells with TRA2A knockdown and negative control cells were subcutaneously injected into the upper-right flank of BALB/c mice(n = 7 in each group). The health status of the mice was monitored daily, while the tumor volume was measured per week. Tumor volume was monitored once a week and determined as follows: (mm^3^) = (Long × Width^2^)/2. After 5 weeks, all mice were euthanized, and tumor tissues were extracted to detect the expression of KI67 and PCNA using immunohistochemical staining. The process of animal experiments was approved by Animal Ethics Committee of Guizhou Medical University (approved number:2,200,044).

### Immunohistochemistry assay

The clinical PC and adjacent tissues were fixed with paraformaldehyde (Servicebio, Wuhan, China), embedded in paraffin (Boster, Wuhan, China), and sectioned into 4 μm thickness. After dewaxing, rehydration, and antigen retrieval with sodium citrate (Servicebio, Wuhan, China), tumor samples were blocked using H_2_O_2_ and 5% bull serum albumin (Servicebio, Wuhan, China) for 30 min at room temperature. The specimens were incubated with primary anti-TRA2A (1:100), KI67 (1:100), anti-PCNA (1:100), and anti-HIF1α (1:100) antibodies for 12 h and horseradish peroxidase-conjugated secondary antibodies (Zsjqbio.biogo; Beijing, China). Next, DAB was used to identify the antigen-antibody complex, and the samples were stained with hematoxylin to visualize the nucleus.

### Chromatin-immunoprecipitation-polymerase chain reaction (ChIP-PCR) assay

PC cells were crosslinked with 1% formaldehyde for 20 min at room temperature. After breaking the DNA into 200–500 bp fragments via ultrasound, Pierce Magnetic ChIP Kit (ThermoFisher Scientific, USA) combined with HIF1α antibody (1:100) or IgG antibody (1:100) was used to enrich the DNA fragments. The purified immunoprecipitated DNA fragments were analyzed using qRT-PCR.

### Statistical analysis

All experiments were performed three times, and the data are shown as the mean ± standard deviation. SPSS 19.0 software (IBM Corp.) was employed to perform all analyses. The difference between two groups was analyzed via Student’s t-test, while one-way exploration of variance (ANOVA) combined with LSD t-test was used to analyze differences between various groups. Co-expression between the two genes was explored using Pearson’s correlation test. *P < 0.05 was regarded as significant.

## Results

Through the analysis of gene expression profiles in GEO, we found that TRA2A expression was upregulated in PC cells under hypoxia. TRA2A expression was higher in PC tissues than in adjacent tissues, as well as in PC cells cultured under hypoxia. High TRA2A expression was associated with advanced stage, poor differentiation, and lymph node metastasis. TRA2A knockdown reduced cell proliferation and mobility under both normoxia and hypoxia as well as reduced PC cell proliferation *in vivo*. Downregulation of TRA2A suppressed the activation of the AKT pathway in both normoxia and hypoxia. HIF1α upregulated the expression of TRA2A by directly binding to its promoter, whereas HIF1α inhibition decreases its expression. TRA2A overexpression reversed the effects of HIF1α knockdown in PC cells.

### TRA2A was recognized as an important hypoxia-associated gene in PC

Gene expression data (GSE9350) containing six normoxic and six hypoxic PC samples were downloaded from the GEO database, and 1446 differentially expressed genes (DEGs) were identified (Figure 1(a)). Additionally, according to the data from TCGA, TRA2A was found to be elevated in PC tissues compared to adjacent tissues (Figure 1(b)). In addition, the expression levels of TRA2A in 48 paired PC tissues and adjacent tissues were determined using RT-PCR and IHC, and both the mRNA and protein levels of TRA2A were found to be elevated in PC tissues (Figure 1(c-d)). Moreover, we observed that high TRA2A expression was associated with advanced stage, poor differentiation, and lymph node metastasis (Table 1). Furthermore, PANC-1 and Capan-2 cells were incubated for 0, 3, 6, and 12 h under hypoxia, and we found that TRA2A expression in PANC-1 and Capan-2 cells gradually increased during hypoxia (Figure 1(e)).

**Figure 1.** TRA2A was identified as a key hypoxia-associated gene in PC. (a) Volcano plot shows the differentially expressed genes in PC cells under normoxia and hypoxia according to gene expression profile GSE9350. (b) The expression of TRA2A in PC tissues and adjacent tissues based on the TCGA and GTEx databases. (c) Quantitative real-time fluorescence PCR was performed to detect the expression of TRA2A in PC tissues and adjacent tissues. (d) Immunohistochemical staining was performed to detect the expression of TRA2A in PC tissues and adjacent tissues. (e) Western blotting was performed to detect the expression of TRA2A in PANC-1 and Capan-2 cells while cultured under hypoxia for 0 h, 3 h, 6 h, and 12 h. *P < 0.05; **P < 0.01.

**Table 1.** The association between TRA2A expression and clinicopathological features of PC patients

TRA2A Expression					
Features	*n*	Low	High	X^2^	P-value
All cases	48	24	24		
Age				0.356	0.551
<60	30	14	16		
≥60	18	10	8		
Gender				0.083	0.773
Man	25	13	12		
Female	23	11	12		
Histological type				0.223	0.637
Adenocarcinoma	43	21	22		
Nonadenocarcinoma	5	3	2		
TNM stage				7.111	0.008
I and II	36	22	14		
III and IV	12	2	10		
Differentiation				5.169	0.023
Well	13	10	3		
Moderate/poor	35	14	21		
Lymph node metastasis				6.701	0.01
No	39	23	16		
Yes	9	1	8		

### Knockdown of TRA2A obviously suppressed PC cell proliferation and mobility under normoxia

Two siRNAs targeted against TRA2A were adopted to suppress the expression of TRA2A under normoxic conditions. The results showed that both effectively inhibited TRA2A expression (Figure 2(a-b)). TRA2A suppression decreased the proliferation of PANC-1 and Capan-2 cells under normoxic conditions at 24 and 48 h (Figure 2(c)). The wound healing (Figure 2(d)) and transwell assays (Figure 2(e)) showed that TRA2A knockdown suppressed the motility of PANC-1 and Capan-2 cells under normoxic conditions.

**Figure 2.** TRA2A knockdown significantly decreased the proliferation and mobility of PC cells under normoxia. (a) qRT-PCR was used to detect the expression of TRA2A while PANC-1 and Capan-2 cells were transfected with si-TRA2A under normoxia. (b) Western blot was used to detect the expression of TRA2A while PANC-1 and Capan-2 cells were transfected with si-TRA2A under normoxia. (c) CCK-8 assay was performed to determine the proliferation rate of si-NC and si-TRA2A group PC cells at 24 h and 48 h under normoxia. (d) Wound healing assay was performed to detect the migration ability while PANC-1 and Capan-2 cells were transfected with si-TRA2A under normoxia. (e) Transwell assay was carried out to determine the invasion ability while PANC-1 and Capan-2 cells were transfected with si-TRA2A under normoxia. *P < 0.05; **P < 0.01.

### *Knockdown of TRA2A inhibited PC cell proliferation* in vivo

The *in vivo* effects of TRA2A knockdown were also determined. We found that tumor tissues with TRA2A knockdown showed a lower growth rate and tumor weight than the negative control (Figure 3(a-c)). We further assessed the expression of KI67 and PCNA in the tumor tissues. The results indicated that KI67 and PCNA expression levels were significantly decreased in the tumor tissues (Figure 3(d)).

**Figure 3.** Inhibition of TRA2A suppressed the proliferation and metastasis of PANC-1 cells *in vivo*. (a) The proliferation rate of tumor cells with TRA2A knockdown and negative control. (b) A typical image of tumor tissues in the negative control and TRA2A knockdown groups. (c) The mean weight of tumor tissues with TRA2A knockdown and negative control. (d) Typical IHC staining images showing KI67 and PCNA expression in transplanted tumors under different experimental conditions.

### Suppression of TRA2A reversed the stimulating effect of hypoxia on PC cell proliferation and motility

PANC-1 and Capan-2 cells were transfected with si-NC, si1-TRA2A, and si2-TRA2A and then cultured under normoxic and hypoxic environments. TRA2A knockdown significantly inhibited TRA2A mRNA and protein levels under hypoxic (Figure 4(a-b)). The CCK-8 assay demonstrated that hypoxia enhanced the proliferation of PANC-1 and Capan-2 cells, whereas TRA2A inhibition reversed the promoting effects of hypoxia on PC cell proliferation (Figure 4(c)). The results of the wound healing assay and transwell experiment showed that PANC-1 and Capan-2 cell migration and invasion were increased under hypoxia, and the inhibition of TRA2A reversed the promoting roles of hypoxia on PC cell migration and invasion (Figure 4(d-e)).

**Figure 4.** Suppression of TRA2A significantly reversed the stimulative effects of hypoxia on the proliferation and mobility of PC cells. (a) qRT-PCR was used to detect the expression of TRA2A while PANC-1 and Capan-2 cells were transfected with si-TRA2A under hypoxia. (b) Western blot was used to detect the expression of TRA2A while PANC-1 and Capan-2 cells were transfected with si-TRA2A under hypoxia. (c) CCK-8 assay was performed to detect the proliferation rate of si-NC and si-TRA2A group PC cells at 24 h and 48 h under hypoxia. (d) Wound healing assay was used to detect the migration ability while PANC-1 and Capan-2 cells were transfected with si-TRA2A under hypoxia. (e) Transwell assay was carried out to determine the invasion ability while PANC-1 and Capan-2 cells were transfected with si-TRA2A under hypoxia. *P < 0.05; **P < 0.01.

### TRA2A activated the AKT pathway in both normoxia and hypoxia

Through GSEA analysis of TRA2A in PC based on the RNA-seq data of TCGA, we found that TRA2A was positively associated with the activation of the AKT pathway (Figure 5(a)). Inhibition of TRA2A under normoxic conditions decreased the expression of p-AKT and increased the expression of PTEN (Figure 5(b)). Hypoxia increased the expression of p-AKT and decreased the expression of PTEN, whereas TRA2A knockdown reversed these effects (Figure 5(c)). These results indicate that TRA2A activates the AKT pathway under both normoxic and hypoxic conditions.

**Figure 5.** TRA2A regulated the AKT pathway. (a) GSEA analysis demonstrated that TRA2A positively regulated the AKT pathway. (b) Western blotting was used to detect the expression of AKT, p-AKT, and PTEN in normoxia after TRA2A knockdown. (c) Western blotting was used to detect the expression of AKT, p-AKT, and PTEN in hypoxia after TRA2A knockdown. *P < 0.05; **P < 0.01.

### TRA2A was a downstream gene of HIF1α

To further investigate the regulatory networks of TRA2A, we analyzed the relationship between TRA2A and HIFs. The motif sequence of HIF1α was obtained from the JASPAR database (Figure 6(a)), and a hypoxia-responsive factor (HRE) site on the TRA2A promoter was predicted (Figure 6(b)). To verify the prediction results, a ChIP assay was performed using an anti-HIF1α antibody in PANC-1 and Capan-2 cells. The results showed that the HRE sequence of the TRA2A promoter was enriched by the anti-HIF1α antibody, and its expression was higher in cells under hypoxia (Figure 6(c)). We found that under hypoxic conditions, the mRNA and protein levels of TRA2A were greatly reduced in HIF1α knockdown PANC-1 and Capan-2 cells, whereas overexpression of HIF1α elevated the mRNA and protein levels of TRA2A (Figure 7(a-b)). In addition, according to data from PC tissues in the TCGA database (R = 0.25, *P* < 0.001; Figure 7(c)) and 48 PC tissues from our research group (R = 0.4079, *P* < 0.001; Figure 7(d-e)), we observed that TRA2A was co-expressed with HIF1α.

**Figure 6.** TRA2A was a target gene of HIF1α. (a) The motif of HIF1α is shown. (b) The hypoxia response element in the promoter of TRA2A is shown. (c) ChIP assays with anti-HIF1α antibody verifying the binding between HIF1α and hypoxia response element of the TRA2A promoter under normoxia and hypoxia. *P < 0.05.

**Figure 7.** TRA2A was co-expressed with HIF1α in PC tissues. (a) qRT-PCR was used to detect the mRNA level of TRA2A while PANC-1 and Capan-2 cells were transfected with si-HIF1α or HIF1α overexpression plasmid under hypoxia. (b) Western blot was used to determine the protein levels of TRA2A while PANC-1 and Capan-2 cells were transfected with si-HIF1α or HIF1α overexpression plasmid under hypoxia. (c) Pearson correlation analysis showed that TRA2A was co-expressed with HIF1α in PC tissues according to the data from the TCGA database. (d) IHC images showing the co-expression of TRA2A and HIF1α. (e) qRT-PCR results showed that TRA2A was co-expressed with HIF1α in our 48 PC tissues. *P < 0.05.

### TRA2A-overexpression reversed the prohibitive roles of HIF1α-suppression on PC cell proliferation and motility under hypoxia

Furthermore, we co-transfected HIF1α siRNA and TRA2A-overexpression plasmid in PANC-1 and Capan-2 cells under hypoxia (Figure 8(a)). The CCK-8 results indicated that HIF1α knockdown suppressed the proliferation of PANC-1 and Capan-2 cells under hypoxia; however, the inhibitory effects of HIF1α knockdown on PANC-1 and Capan-2 proliferation (Figure 8(b)) were reversed by TRA2A-overexpression. Similarly, according to wound healing and transwell assays, HIF1α suppression greatly reduced the migration and invasion of PANC-1 and Capan-2 cells under hypoxia, whereas overexpression of TRA2A in HIF1α knockdown cells reduced the inhibitory effects of HIF1α knockdown on PANC-1 and Capan-2 migration and invasion (Figure 8(c-d)).

**Figure 8.** Overexpression of TRA2A reversed the inhibitory effects of HIF1α knockdown on PC cell proliferation and mobility under hypoxia. PANC-1 and Capan-2 cells were divided into four groups as follows: si-NC + vector, si-HIF1α + vector, si-NC + Lv-TRA2A and si-HIF1α + Lv-TRA2A. All group cells were cultured in hypoxia. (a) Western blot was used to detect the expression of TRA2A and HIF1α in each group cells. (b) CCK-8 assay was performed to detect the proliferation rate of each group of cells at 24 h and 48 h. (c) Wound healing assay was used to detect the migration ability while each group of cells. (d) Transwell assay was carried out to determine the invasion ability while each group of cells. *P < 0.05; **P < 0.01.

## Discussion

Hypoxia is commonly observed in the solid tumor microenvironment, including PC. The proliferation and metastasis of tumor cells can be promoted by hypoxia [19]. Several hypoxia-related genes have been shown to play roles in hypoxia. However, the molecular mechanism underlying hypoxia regulation in PC remains unclear.

In the present study, using bioinformatics, TRA2A in PC cells was found to be upregulated in hypoxia compared with normoxia. TRA2A was also upregulated in PC tissues compared with adjacent tissues, and was associated with poor clinical traits. Through related experiments, we confirmed the increase in TRA2A expression in PC cells and PC tissues cultured under hypoxia. Therefore, TRA2A was considered to be a key hypoxia-related gene that may drive PC progression.

Previous studies on the expression of TRA2A and its significance have been extensive. Xu et al. confirmed that high expression of TRA2A indicates poor prognosis in patients with hepatocellular carcinoma [20]. Sanchez et al. found that TRA2A is a biomarker for the development of prostate cancer [21]. Liu et al. showed that TRA2A promotes taxol resistance and tumor progression in patients with triple-negative breast cancer [15]. Nevertheless, the biological role of TRA2A in PC cells under normal and anoxic conditions remains unclear. In this study, TRA2A knockdown greatly inhibited the proliferation and migration of PC cells under normoxic and hypoxic conditions. It was proved that TRA2A acts as an oncogene in PC and is associated with hypoxic environments.

AKT signaling is a key factor involved in the etiology of PC and is commonly activated in PC. Activation of AKT signaling contributes to PC cell proliferation, metastasis, and differentiation [22,23]. Previous studies have indicated that hypoxia is a key driving force that enhances the activation of AKT signaling [24]. For example, hypoxia enhances the activation of AKT in PC cells by LIM zinc finger domain containing 1 and promotes the progression of PC [25]. The interleukin-8 forms a feedback loop with AKT and HIF1α, thus continuously increasing PC cell proliferation and metastasis under hypoxia [26]. However, the mechanisms underlying the activation of AKT under hypoxic conditions in PC are largely unknown. In the current study, we found that TRA2A could activate the AKT pathway in normoxia and hypoxia. Therefore, TRA2A may be a key factor in the regulation of AKT signaling.

Hypoxia exerts a significant effect on many cancers, and hypoxia-inducible elements are key mediators of hypoxia reactions [27]. HIFs, such as HIF1α, HIF2α, and HIF3α, binds to the target gene promoter to promote its transcription, thus accelerating cancer cell migration, proliferation, and invasion [28]. In recent years, some downstream genes of HIFs have been identified. For instance, Wang et al. showed that HIF1α promotes metastasis in hepatocellular carcinoma by promoting the expression of lysine oxidase 2 in hypoxic environments [29]. Similarly, TUFT1 regulates metastasis in pancreatic cancer through epithelial-mesenchymal transformation induced by HIF1-Snail [30]. In this study, we found that HIF1α directly binds to the TRA2A promoter and regulates its expression. TRA2A overexpression reversed the effects of HIF1α knockdown on the biological functions of PC cells. Interestingly, TRA2A overexpression also increased the expression of HIF1α. As p-AKT has the potential to regulate the stability of HIF1α, we considered that TRA2A upregulated the expression of HIF1α by mediating the activation of AKT signaling. This evidence indicates that TRA2A may be a key target of HIF1α, and a TRA2A/AKT/HIF1α positive feedback loop may exist in PC cells.

## Conclusion

TRA2A is a core target gene of HIF1α, which has the potential to drive the proliferation and mobility of PC cells by mediating the activation of the AKT pathway.

## Supplementary Material

Supplemental Material
